# Effect and Mechanism of Lidocaine Pretreatment Combined with Dexmedetomidine on Oxidative Stress in Patients with Intracranial Aneurysm Clipping

**DOI:** 10.1155/2021/4293900

**Published:** 2021-11-24

**Authors:** Junting Zhang, Hongwei Zhang, Liang Zhao, Zhanqi Zhao, Ying Liu

**Affiliations:** Department of Anesthesiology, The Third Affiliated Hospital of Qiqihar Medical College, Qiqihar 161000, China

## Abstract

This study aimed to explore the effect and mechanism of lidocaine pretreatment combined with dexmedetomidine on oxidative stress in patients with intracranial aneurysm clipping. Many studies have used various drugs such as lidocaine to explore the effect and mechanism of lidocaine pretreatment. A total of 80 patients with intracranial aneurysm clipping surgery were randomly divided into 4 groups: the single lidocaine group, single dexmedetomidine group, lidocaine combined with dexmedetomidine group, and control group. The thread embolism method was used to establish a stable intracranial aneurysm model of Hashimoto rats. Fifty adult rats were randomly divided into a sham operation group, ligation of the left common carotid artery and bilateral posterior branch of renal artery, lidocaine group, dexmedetomidine group, and lidocaine combined with dexmedetomidine group. The colorimetric method was used to determine the oxidative stress indicators in brain tissue: MDA content, SOD activity, and T-AOC content. The western blot method characterized the protein levels related to oxidative stress: nNOS, iNOS, and NADPH oxidase subunits p22phox, gp91phox, and p47phox. The differences in each index between the groups were statistically significant (*P* < 0.05). Animal experiment results revealed that the content of MDA in the brain tissue of rats in the LD group was significantly lower than that in the single-drug group and sham group. The T-AOC and SOD concentrations in the LD group were significantly higher than those in the single-drug group and sham group, and the differences between the groups were statistically significant (*P* < 0.05). The protein expression of the LD group was significantly lower than that of the drug-alone group and model group, and the difference between groups was statistically significant (*P* < 0.05). To sum up, lidocaine pretreatment combined with dexmedetomidine can effectively maintain the hemodynamic stability of patients with intracranial aneurysm clipping and reduce postoperative oxidative stress response. Its mechanism of action may be related to the inhibition of oxidative stress damage mediated by nNOS, iNOS, and p22phox, gp91phox, and p47phox in the hippocampus. Our study has significant and applicable medical aspects in lidocaine pretreatment combined with dexmedetomidine on oxidative stress in patients.

## 1. Introduction

Intracranial aneurysm clipping is one of the common surgical procedures for the treatment of cerebral aneurysms. Several clinical studies have proved that the serial processes of neurosurgery and anesthesia can cause oxidative stress in the body [1–3]. Brain tissue is sensitive to oxidative stress. Oxidative stress injury is an important cause of cerebral ischemia injury [4] and plays a vital role in each link in the acute stage of ischemic cerebrovascular disease. Therefore, it is crucial to select pharmacologically effective cerebral protective drugs during craniocerebral surgery to improve the stability of intraoperative cerebral blood supply dynamics and oxidative stress levels in patients and to reduce the damage caused by cerebral ischemia.

According to the research report, lidocaine is an aminoamide anesthetic. As an anesthetic drug in clinic, it can reduce the intracellular Na^+^ and Ca^2+^ concentration and suppress the outflow of k^+^, inhibit the release of oxygen free radicals by neutrophils, and increase the survival number of CA_1_ pyramidal neurons [5, 6]. Therefore, it inhibits oxidative stress induced by brain injury and stimulation, and endotoxin plays a protective role in brain tissue and nerve cells [7, 8]. Intravenous lidocaine can also effectively alleviate blood flow fluctuations during surgical anesthesia, especially during anesthesia induction intubation and recovery period. It reduces stress response, significantly improves neurological deficits after ischemia, and reduces brain histomorphology damage after ischemia.

Studies have revealed that catecholamine level increases in patients with craniocerebral injury after operation, and it is of great significance to regulate sympathetic nerve cells to maintain stable hemodynamics [9]. Dexmedetomidine is an effective and highly selective adrenoceptor *α*2 receptor agonist in locus coeruleus that modulates norepinephrine levels to achieve good sedative and hypnotic effects. It can produce effects in the posterior horn of the spinal cord to achieve anti-injurious effects and produce effects in the periphery and center to achieve antisympathetic activity [10]. Studies have shown that dexmedetomidine can alleviate the harmful stimulation caused by surgery, maintain cardiovascular stability, and reduce cerebral blood flow during the operation of craniocerebral patients [11]. Furthermore, dexmedetomidine can reduce the level of inflammatory factors in patients with craniocerebral injury. It improves cerebral oxygen metabolism, reduces oxidative stress reaction, and effectively improves the stability of central blood vessels in craniocerebral operation. It also reduces brain edema caused by craniocerebral injury [12], thus improving the ischemic and hypoxic injury of brain tissue with effect [13].

However, there are few studies on the effects of dexmedetomidine combined with lidocaine on oxidative stress response of patients undergoing intracranial aneurysm clipping. It is not clear whether the combination of dexmedetomidine and lidocaine has a synergistic effect. Therefore, in this study, dexmedetomidine combined with lidocaine-assisted anesthesia was given to patients with craniocerebral injury who were undergoing emergency surgery in our hospital for a certain period. Its effect on oxidative stress reaction of patients was studied. On this basis, the mechanism of lidocaine and dexmedetomidine affecting oxidative stress response is the key issue of this paper.

## 2. Materials and Methods

### 2.1. Materials

Total superoxide dismutase (SOD test kit), the T-AOC kit, and the MDA detection kit were from Oubei Biotechnology Co., Ltd., Beijing. The BCA protein concentration determination kit and cell lysate were from Beyotime, Shanghai. Rabbit internal reference monoclonal antibody GAPDH (item number: AF1186), rabbit anti-mouse monoclonal antibodies nNOS (item number: AF1819), iNOS (item number: AF7281), mouse anti-human gp91phox monoclonal antibody (item number: AF2290), and other antibodies were purchased from Beyotime, Beijing. Rabbit anti-human polyclonal antibodies p22phox (item no. 66020-1-lg), p47phox (item number 28187-1-AP), horseradish peroxidase-labeled goat anti-rabbit IgG, and horseradish peroxidase-labeled goat anti-mouse IgG were purchased from Proteintech. The PVDF blotting membrane was purchased from BBI Biotech, USA.

### 2.2. Methods

#### 2.2.1. Clinical Sample Collection and Data

From June 2018 to December 2019, a total of 80 patients undergoing intracranial aneurysm clipping in the Third Affiliated Hospital of Qiqihar Medical College were recruited for clinical study. There was no statistical difference in general data such as gender, age, weight, or ASA classification in patients, nor there were patients with a history of hepatic or renal insufficiency or allergy to narcotic drugs. All included patients met the diagnostic criteria of intracranial aneurysms and American Society of Anesthesiologists (ASA) grade I-II. Patients with severe cardiopulmonary, liver or kidney injury, abnormal coagulation function, respiratory or circulatory diseases, or with allergy to drugs applied in this study were excluded. In this study, all patients and their families were informed and signed informed consent forms. This study was approved by the Ethics Committee. The abovementioned patients were randomly divided into four groups (20 cases in each group): the lidocaine group (L group), dexmedetomidine group (D group), lidocaine combined with dexmedetomidine group (LD group), and control group (A group). Patients in the D group were infused with dexmedetomidine 1 *μ*g/kg × 15 min during operation and then pumped at the rate of 0.55 *μ*g/kg^−1^∙h^−1^ until the end of operation. Patients in the L group were given intravenous injection of 2% lidocaine 1.5 mg/kg at the rate of 2 mg/kg^−1^∙h^−1^ during operation. The drug usage in the LD group was the same as that in the L group and D group. Patients in group A were given 0.9% saline equal to the abovementioned groups. See Table 1 for details.

#### 2.2.2. Clinical Outcome Measures

The levels of heart rate (HR) and mean arterial pressure (MAP) were monitored and recorded before operation (T_0_), at the beginning of tumor-bearing artery occlusion (T_1_), at the end of tumor-bearing artery occlusion (T_2_), at the end of operation (T_3_), and 24 h after operation (T_4_). Besides, the elbow venous blood was collected from the four groups of patients at the abovementioned time points, and the superoxide dismutase (SOD) activity, malondialdehyde (MDA) level, serum S-100*β* protein content, and neuron-specific enolase (NSE) level were determined.

#### 2.2.3. Experimental Animals and Grouping

The rat model of intracranial aneurysm was established by the thread embolism method: 50 adult SD rats weighing (200 ± 20) g were ligated in the left common carotid artery and the posterior branches of bilateral renal arteries. They were randomly divided into 5 groups (*n* = 10): the sham operation group (sham group, rats were given the same amount of normal saline), ligation of left common carotid artery and posterior branches of bilateral renal arteries (model group, rats were the same amount of normal saline during operation), lidocaine group (L group, rats were injected with 2% lidocaine 1.5 mg/kg intravenously during operation), dexmedetomidine group (D group, rats were given dexmedetomidine 1 *μ*g/kg), and the two drugs combined group (LD group, the same as L group and D group).

#### 2.2.4. Collection and Treatment of Specimens

The rats were fasted for 12 h after operation, then anesthetized, and decapitated. Six rats were taken from each group, and 1 g of aneurysm and surrounding tissues were homogenized and centrifuged (4000 r/min) × 10 min to obtain the supernatant for later use. The left hippocampus was preserved at −80°C for western blot experiment.

#### 2.2.5. Determination of MDA, T-AOC Content, and SOD Activity in Rat Brain Tissue

The MDA content and SOD activity were detected with MDA and SOD kits. The colorimetric method was used to determine the oxidative stress indicators in brain tissues of MDA content, SOD activity, and T-AOC content. The activity of SOD was determined by the WST method, the content of MDA by the TBA method, and the activity of T-AOC by the Fe^3+^ reduction method.

#### 2.2.6. Western Blot Method in Detecting Protein Expression

The expression of oxidative stress-related proteins in each group was detected by western blot, including nNOS, iNOS, and NADPH oxidase subunits p22phox, gp91phox, and p47phox, and internal reference GAPDH. The frozen tissue proteins mentioned above were extracted by lysis on ice, and the protein concentration was determined by the BCA method. The sodium dodecyl sulfate-polyacrylamide gel electrophoresis (SDS-PAGE) was applied for western blot experiment. The immune reaction of polyclonal antibodies GAPDH (1 : 1000), p22phox and p47phox (1 : 500), and monoclonal antibodies nNOS and iNOS (1 : 200) were determined with highly sensitive enhanced chemiluminescence.

### 2.3. Statistical Treatment

All data were statistically processed using SPSS 17.0 software and expressed as $\bar{x}\pm s$. Comparisons between sample means were performed by the *t*-test, and *P* < 0.05 or *P* < 0.01 was statistically significant.

## 3. Results

### 3.1. Hemodynamic Indexes

There was no significant difference in HR and MAP levels between the four groups at T_0_ (*P* > 0.05). At T_1_, T_2_, T_3_, and T_4_, the HR and MAP levels in each group were listed as follows: A group > D group > L group > LD group (*P* < 0.05), as shown in Figures 1 and 2.

### 3.2. Evaluation of Oxidative Stress Level

There were differences in the concentrations of S-100*β* protein, NSE, SOD, and MDA at different time points in each group. All the four groups showed elevated concentrations at T_2_ than T_1_ (*P* < 0.05) and decreased concentrations at T_3_ than T_2_, with significant differences among the four groups (*P* < 0.05).

At T_0_, there was no significant difference in serum SOD, MDA, S-100*β* protein, and NSE among the four groups (*P* > 0.05). From T_1_ to T_4_, the concentration of S-100*β* protein, MDA, and NSE in serum was listed as follows: A group > D group > L group > LD group, and the concentration of SOD was as follows: A group < D group < L group < LD group, with significant differences among groups (*P* < 0.05). The details are shown in Figure 3. It can be seen that lidocaine and dexmedetomidine can reduce the concentrations of serum S-100*β*, NSE, and MDA and enhance SOD activity, and the combined application of the two drugs can significantly alleviate the level of oxidative stress.

### 3.3. Effects of MDA, T-AOC Content, and SOD Activity in Rat Brain Tissue

Compared with the Sham group, MDA content in brain tissue of rats in the L group, D group, and LD group significantly increased (*P* < 0.05), while T-AOC content and SOD activity significantly decreased (*P* < 0.05). Compared with the model group, MDA content in brain tissue of rats in L, D, and LD groups significantly decreased (*P* < 0.05), while T-AOC content and SOD activity significantly increased (*P* < 0.05). Compared with the LD group, the content of MDS in the L group and D group was markedly higher (*P* < 0.05), and the activities of T-AOC and SOD were markedly lower (*P* < 0.05). MDA content: sham group > D group > L group > LD group > model group; T-AOC and SOD concentrations: sham group < D group < L group < LD group < model group. More details are shown in Figure 4. According to the abovementioned animal experiment results, both lidocaine and dexmedetomidine can improve the oxidative stress level of rats, and the synergistic effect of the two drugs can significantly enhance the effect.

### 3.4. Analysis of Western Blot Results

Compared with the sham group, the expression levels of nNOS, iNOS, and p22phox, p91phox, and p47phox in brain tissue of rats in other groups were significantly higher (*P* < 0.05), showing a relatively high level of oxidative stress. Compared with the A group, the expression of nNOS, iNOS, p22phox, p91phox, and p47phox protein in the rat brain was reduced to varying degrees in the L group, D group, and LD group (*P* < 0.05), and LD group shows stronger inhibitory effect, as shown in Figure 5. This conclusion is consistent with the previous research results, suggesting that lidocaine and polymetamidine have a synergistic effect, which can inhibit the oxidative stress injury mediated by nNOS, iNOS, and p22phox, p91phox, and p47phox proteins, and then play a protective role in the process of intracranial aneurysm clipping.

## 4. Discussion

The surgical procedure of aneurysm clamping is prone to cause brain tissue and nerve cell damage in patients, so perioperative brain protection has become a research concern [14–16]. Studies [17, 18] have shown that lidocaine is an effective brain protection drug in clinic, which can inhibit the release of oxygen free radicals and reduce the risk of cerebral ischemia-oxygen injury during operation. Dexmedetomidine is used in surgery for anesthesia to effectively maintain the smoothness of perioperative hemodynamic parameters, thereby reducing neurological damage to the patient's brain tissue [19–21]. Both of the abovementioned drugs show a certain brain protection effect, but whether the two drugs are used together has synergistic effect and synergistic effect of brain protection, and the related mechanism of action is rarely reported.

According to this study, compared with those receiving normal saline, patients who received lidocaine or dexmedetomidine lone during the operation had lower HR and MAP levels from T_1_ to T_4_, showing a relatively stable trend. The group adopting lidocaine combined with dexmedetomidine showed more obvious advantages. Studies have shown that the combination of the two drugs can effectively reduce the adverse effects of surgery on patients' respiratory system and body circulation and improve perioperative hemodynamic stability.

S-100*β* protein and NSE are marker proteins of brain tissue injury. Increased content of S100*β* protein in serum indicates a serious trend of nerve injury [22–24]. NSE is the marker enzyme of neuron injury [25], and the concentration of NSE in blood reflects the degree of brain injury in patients [26, 27]. When craniocerebral injury occurs, a large number of oxygen free radicals are produced in the body, which increases the content of MDA and impairs cell function [28, 29]. SOD is a powerful antioxidant enzyme in the body, which can remove free radicals and effectively relieve lipid peroxidation damage during cerebral ischemia [30, 31]. Therefore, in this study, the abovementioned four indexes were observed at each time point of clamping operation, and the effects of combined application of lidocaine and dexmedetomidine on the oxidative stress level of patients were evaluated. It was found that the serum S-100*β* protein, NSE level, and MDA concentration of patients in the L group, D group, and LD group were significantly lower than those in the A group, and the SOD content was significantly higher than that in the A group. More importantly, the LD group showed the most significant regulatory effect, indicating superior ability to improve oxidative stress level. To sum up, lidocaine combined with dexmedetomidine can effectively reduce the oxidative stress reaction of perioperative patients, reduce the degree of brain injury, and play a more effective role in brain protection.

In order to verify the reaction mechanism of the abovementioned research, rat intracranial aneurysm models were established, and the levels of SOD, T-AOC, and MDA in the brain tissue of experimental rats, as well as the changing trend of nNOS, iNOS, and p22phox, p91phox, and p47phox protein expression levels, were detected for verification. The contents of SOD, T-AOC, and MDA in the body reflect the metabolic level of oxygen free radicals in the body. The animal experiment of this study indirectly reflects the oxidative stress state of model rats by measuring the changes of the contents of the three. The results showed that lidocaine and dexmedetomidine can improve the oxidative stress level of rats by inducing the changes of SOD activity, T-AOC, and MDA content, and the two drugs have a synergistic effect, which can more strongly improve the oxidative stress state. This further confirms the conclusion of previous research.

Then, we assessed the expression of oxidative stress indicators of nNOS, iNOS, and NADPH oxidase subunits p22phox, p91phox, and p47phox in rat brain tissue and then discussed the possible mechanism of lidocaine combined with dexmedetomidine in inhibiting oxidative stress. The animal experiments showed that the expressions of nNOS, iNOS, and p22phox, p91phox, and p47phox in the L group, D group, and LD group were decreased, and these levels in the LD group were significantly lower than those in the L group and D group. The abovementioned results indicated that lidocaine pretreatment combined with dexmedetomidine can effectively improve the oxidative stress injury induced by NADPH oxidase, nNOS, and iNOS via decreasing the expression of related proteins.

## 5. Conclusions

However, there are still some limitations in our study, and we need to conduct a deeper study about lidocaine and dexmedetomidine in future work. In our research work, we found that lidocaine and dexmedetomidine have a synergistic effect, which can improve the perioperative hemodynamic stability of patients with intracranial aneurysm clipping. The inhibitory effect of the combination of the two drugs on the oxidative stress level of the body was further verified in rat models. Besides, the drugs can improve the level of oxidative stress by regulating the expression of oxidative stress-related proteins, so as to achieve the purpose of perioperative protection of craniocerebral injury.

## Figures and Tables

**Figure 1:** Comparison of HR at each time point in the four groups of patients. There are significant differences between groups, ^*∗*^*P* < 0.05.

**Figure 2:** Comparison of MAP at each time point in the four groups of patients. There are significant differences between groups, ^*∗*^*P* < 0.05.

**Figure 3:** Comparison of blood S-100*β*, NSE, SOD, and MDA levels in four groups of patients at different time points. (a) Blood S-100*β*, (b) NSE, (c) SOD, and (d) MDA. There are significant differences between groups, ^*∗*^*P* < 0.05.

**Figure 4:** Comparison of the concentrations of MDA (a), T-AOC (b), and SOD (c) in the brain tissue of rats in each group. There are significant differences between groups, ^*∗*^*P* < 0.05.

**Figure 5:** Western blotting results. (a) Western blotting is used to detect the protein expressions of nNOS, iNOS, and p22phox, p91phox, and p47phox in rat brain tissues; (b) histogram of the relative protein gray values in (a). There are significant differences between groups, ^*∗*^*P* < 0.05, ^*∗∗*^*P* < 0.01.

**Table 1:** Comparison of general data of the four groups of patients (*n* = 20, $\bar{x}\pm s$).

Group	Age (years)	Weight (kg)	ASA classification	Operation time (min)
Group A	57 ± 4	63 ± 2	6/13	302 ± 15
Group D	56 ± 5	62 ± 3	5/11	306 ± 17
Group L	59 ± 7	62 ± 3	6/12	303 ± 20
Group LD	57 ± 6	64 ± 2	7/12	304 ± 14

## Data Availability

The datasets used and/or analyzed during the present study are available from the corresponding author on reasonable request.

## References

[1] Yu J.-M., Sun H., Wu C., Dong C.-S., Lu Y., Zhang Y. (2016). The analgesic effect of ropivacaine combined with dexmedetomidine for incision infiltration after laparoscopic cholecystectomy. *Surgical Laparoscopy Endoscopy & Percutaneous Techniques*.

[2] Miki K., Yoshioka T., Hirata Y. (2016). Surgical outcome of acute and subacute subdural hematoma with endoscopic surgery. *Noshinkeigeka*.

[3] Zeng Y., Xu D., Wei J. (2021). Lidocaine pretreatment up-regulates aquaporin-5 expression in primary alveolar epithelium type II cells injured by lipopolysaccharides. *Pakistan journal of pharmaceutical sciences*.

[4] Kawata R., Terada T., Lee K., Higashino M., Ichihara S. (2016). Surgical management for benign parotid tumors: review of a 16-year experience with 633 patients. *Nippon Jibiinkoka Gakkai Kaiho*.

[5] Bekker A., Sturaitis M., Bloom M. (2008). The effect of dexmedetomidine on perioperative hemodynamics in patients undergoing craniotomy. *Anesthesia & Analgesia*.

[6] Li Y., Zeng M., Chen W. (2014). Dexmedetomidine reduces isoflurane-induced neuroapoptosis partly by preserving PI3K/akt pathway in the Hippocampus of neonatal rats. *PLoS One*.

[7] Lewartowska N. D., Skotnickak G. (2016). Minor head trauma-trivial matter or sirious diagnostic and therapeutic problem: the role of Infrascanner in the diagnostic process. *Dev Period Med*.

[8] Jin Y., Jiang J., Zhang X. (2016). Effect of reflection of temporalis muscle during cranioplasty with titanium mesh after standard trauma craniectomy. *Journal of Craniofacial Surgery*.

[9] Kim S.-K., Song M.-H., Lee I.-J., Lee J.-H., Choi I.-C. (2016). Dexmedetomidine for sedation in pediatric patients who received more than 20 sessions of radiation therapy: two cases report. *Korean Journal of Anesthesiology*.

[10] Gupta K., Rastogi B., Gupta P. K., Singh I., Singh V. P., Jain M. (2016). Dexmedetomidine infusion as an anesthetic adjuvant to general anesthesia for appropriate surgical field visibility during modified radical mastectomy with i-gel: a randomized control study. *Korean Journal of Anesthesiology*.

[11] Kim J. K. (2016). An introduction to the various role of dexmedetomidine. *Korean Journal of Anesthesiology*.

[12] Zhao P., Zhou R., Zhu X.-Y. (2015). Matrine attenuates focal cerebral ischemic injury by improving antioxidant activity and inhibiting apoptosis in mice. *International Journal of Molecular Medicine*.

[13] Zhang T. Z., Zhou J., Jin Q. (2014). Protective effects of remifentanil preconditioning on cerebral injury during pump-assisted coronary artery bypass graft. *Genetics and Molecular Research*.

[14] Lvovskaya E. I., Derginskyi N. V., Sadova V. A., Symnaya D. B. (2016). Prognostic value of the parameters of free radical oxidation in traumatic brain injury. *Biomeditsinskaya Khimiya*.

[15] Sonawane N., Balavenkatasubramanian J., Gurumoorthi P., Jadhav P. (2016). Quality of post-operative analgesia after epidural dexmedetomidine and ketamine: a comparative pilot study. *Indian Journal of Anaesthesia*.

[16] Saichan X., Wei C., Qinglong F., Jun W., Lei X. (2016). Plasma cortisol as a noninvasive biomarker to assess severity and prognosis of patients with craniocerebral injury. *European Review for Medical and Pharmacological Sciences*.

[17] Tang Y. K., Shi M., Ou G. S., Zhao H. (2014). Role of acute alcohol poisoning and craniocerebral trauma in the mechanism of death caused by subarachnoid hemorrhage. *Fa Yi Xue Za Zhi*.

[18] Akdemir H., Yardan T., Kati C. (2014). The role of S100B protein, neuron-specific enolase, and glial fibrillary acidic protein in the evaluation of hypoxic brain injury in acute carbon monoxide poisoning. *Human & Experimental Toxicology*.

[19] Macedo R. C. d., Tomasi C. D., Giombelli V. R. (2013). Lack of association of S100*β* and neuron-specific enolase with mortality in critically ill patients. *Revista Brasileira de Psiquiatria*.

[20] Van L. J., Wain M. S. (2003). The Janus face of glial-derived S100*β*: neficial and detrimental functions in the brain. *Restorative Neurology and Neuroscience*.

[21] Lei B., Popp S., Capuano-Waters C., Cottrell J. E., Kass I. S. (2004). Lidocaine attenuates apoptosis in the ischemic penumbra and reduces infarct size after transient focal cerebral ischemia in rats. *Neuroscience*.

[22] Arsalani-Zadeh R., Ullah S., Khan S., MacFie J. (2011). Oxidative stress in laparo-scopic versus open bdominalsurgery: a systematic review. *Journal of Surgical Research*.

[23] Geze S., Cekic B., Imamoğlu M. (2012). Use of dexmedetomidine to prevent pulmonary injury after pneumoperitoneum in ventilated rats. *Surgical Laparoscopy Endoscopy & Percutaneous Techniques*.

[24] Su S., Li Q., Liu Y. (2014). Sesamin ameliorates doxorubicin-induced cardiotoxicity: i. *Toxicology Letters*.

[25] Zhang J.-x., Yang J.-r., Chen G.-x. (2013). Sesamin ameliorates arterial dysfunction in spontaneously hypertensive rats via downregulation of NADPH oxidase subunits and upregulation of eNOS expression. *Acta Pharmacologica Sinica*.

[26] Li W.-x., Kong X., Zhang J.-x., Yang J.-r. (2013). Long-term intake of sesamin improves left ventricular remodelling in spontaneously hypertensive rats. *Food Funct.*.

[27] Ueno M., Sakamoto H., Tomimoto H. (2004). Blood-brain barrier is impaired in the hippocampus of young adult spontaneously hypertensive rats. *Acta Neuropathologica*.

[28] Kishi T., Hirooka Y., Sunagawa K. (2012). Telmisartan protects against cognitive decline via up-regulation of brain-derived neurotrophic factor/tropomyosin-related kinase B in hippocampus of hypertensive rats. *Journal of Cardiology*.

[29] Jiang T., Gao L., Shi J., Lu J., Wang Y., Zhang Y. (2013). Angiotensin-(1-7) modulates renin-angiotensin system associated with reducing oxidative stress and attenuating neuronal apoptosis in the brain of hypertensive rats. *Pharmacological Research*.

[30] Wang Z. X., Huang C. Y., Hua Y. P., Huang W. Q., Deng L. H., Liu K. X. (2014). Dexmedetomidine reduces intestinal and hepatic injury after hepatectomy with inflow occlusion under general anaesthesia: a randomized controlled trial. *British Journal of Anaesthesia*.

[31] Liang C., Cang J., Wang H., Xue Z. (2013). Propofol attenuates cerebral ischemia/reperfusion injury partially using heme oxygenase-1. *Journal of Neurosurgical Anesthesiology*.

